# The Construction of Folk Sports Featured Towns Based on Intelligent Building Technology Based on the Internet of Things

This article has been retracted.

**DOI:** 10.1155/2022/4541533

**Published:** 2022-01-25

**Authors:** Zhou Li-yun, Wang Cheng-ke, Zhang Qiang

**Affiliations:** ^1^Guangxi Normal University of Nationalities, Guangxi, Chongzuo 532200, China; ^2^Guangxi College for Preschool Education, Guangxi, Nanning 530000, China; ^3^Guangxi Institute of Technical, Guangxi, Chongzuo 532200, China

## Abstract

With the emergence of the Internet of Things, technology and Internet thinking have entered traditional communities, and combined with traditional technologies, many new and better management methods and solutions have been born. Among them, the concept of intelligent buildings is also known to people. Based on big data technology, cloud computing technology, and Internet of Things technology, smart buildings provide smart and convenient devices and services for smart device users. The Internet of Things technology is entering our lives at an unimaginable speed. It has been applied in many fields. Smart home, smart transportation, smart medical, smart agriculture, and smart grid are widely used in the Internet of Things technology. The application of Internet of Things technology to the construction of folk sports characteristic towns is of great significance. The construction of folk sports characteristic towns and the protection of intangible cultural heritage have the same purpose and interoperability of elements as the development of traditional cities. From the perspective of protecting folk culture and intangible cultural heritage, it is effective to promote the development of small towns with folk custom characteristics. Based on the research on the construction of folk-custom sports towns, this paper proposes a series of data model analysis and analyzes the proportion of sports preferences in the survey of volunteers in the folk-custom sports towns. The final result of the research shows that the ball games sports personnel accounted for the largest proportion, with 156 people accounting for 48.15%. This shows that about half of the people like ball sports, which proves that ball sports should be the mainstay of folk sports towns, and other sports should be supplemented by other sports.

## 1. Introduction

With the economic growth and the improvement of living standards, the influence of sports in the world is increasing, and people's pursuit of physical exercise is gradually increasing. Therefore, it is very promising to build a small town with folk sports characteristics. Incorporate into the town, and connect the network, things, and places where people live and even cities to the network through the Internet of Things, and finally control them through the use of the “Internet of Things”. However, the premise of all this is the existence of the Internet. Therefore, in recent years, the Internet has developed rapidly and has entered thousands of households, allowing the Internet of Things to be used and developed. The Internet of Things has played a key role in national construction and development. The Internet of Things refers to the real-time collection of any object or process that needs to be monitored, connected, and interactive through various devices and technologies such as information sensors, radio frequency identification technology, global positioning system, infrared sensors and laser scanners, and the collection of various required information such as sound, light, heat, electricity, mechanics, chemistry, biology, and location, which can be accessed through various possible networks, realize the ubiquitous connection between things and people, and realize the intelligent perception, identification, and management of goods and processes. The Internet of Things is an information carrier based on the Internet and traditional telecommunication networks. It allows all ordinary physical objects that can be independently addressed to form an interconnected network.

In recent years, in the research of intelligent building technology combined with folk sports characteristic towns, many researchers have conducted research on it and achieved good results. For example, Zhou and Zhang believe that folk culture is the carrier of intangible cultural heritage. Intangible cultural heritage has the attributes of “intangible” and “intangible,” which makes it strictly different from material cultural heritage. Folk culture complements each other, and they are closely related to some extent [1, 2]. Zhang and Yuan believe that the difference between smart buildings and traditional buildings is that they are composed of wireless communication, automation, etc. Smart buildings are no longer just a building body; it is an online “life body” with self-learning, self-perception, and self-processing. The function of sensing, processing, and learning information [3]. At present, there are many researches on the construction of folk custom sports under the intelligent building technology. These predecessors' theories and experimental results provide a theoretical basis for the research of this article. [4–7] “The Internet of things is the Internet connected with things.” This has two meanings: first, the core and foundation of the Internet of Things are still the Internet, which is an extended and extended network based on the Internet. Second, its client extends and extends to any goods and goods for information exchange and communication. Therefore, the definition of the Internet of Things is to connect any item to the Internet through information sensing equipment such as RFID, infrared sensor, global positioning system, and laser scanner according to the agreed protocol [8–13].

Based on the analysis of the construction of folk sports characteristic towns under the intelligent building technology of the Internet of Things, this paper elaborates on the relevant design concepts of folk towns. The town's material and cultural space are arranged, and in the subsequent tourism development and operation, the relevant information on the integration of folk customs and sports will be continuously disseminated to the outside world [14–17]. To make villagers in folk sports characteristic towns break away from traditional agricultural production-based lifestyles, carry out industrial upgrades, make them truly carriers of intangible cultural heritage, build the environment of folk sports characteristic towns, and protect and spread the wealth of folk culture. The basic characteristics of the Internet of Things from the perspective of communication objects and processes and the information interaction between things, people, and things are the core of the Internet of Things. The basic characteristics of the Internet of Things can be summarized as overall perception, reliable transmission, and intelligent processing. The function of obtaining information. It mainly refers to the perception and recognition of information. Information perception refers to the perception and sensitivity to the attribute state and its change mode of things. Information recognition refers to the ability to express the state of things in a certain way [18–20].

## 2. The Intelligent Design Viewpoint and Design Significance of the Folk Sports Characteristic Town

### 2.1. Viewpoints on the Design of Featured Folk Sports Towns

#### 2.1.1. Comprehensive Correlation between the Various Subsystems

The various subsystems of the intelligent building are not the same on the surface, and the names are different, but in terms of structure, we can find common connections between them, and some functions of each subsystem can be shared with each other. According to the concept of the Internet of Things, a three-layer architecture model can be removed for each subsystem, namely, the detection layer, the transmission layer, and the application layer. The intelligent building industry often refers to this structure as front-end, transmission, and back-end. The video surveillance system monitor belongs to the detection layer, and the signal transmission path belongs to the transmission layer; the video surveillance platform, storage system, operating keyboard, and wall control system belong to the application layer; the card reader access card, door sensor, and access control system belong to the application layer. The feedback signal and output button of the access control lock system belong to the detection level, the shielded cable signal transmission path belongs to the application level, and the access control system server belongs to the application layer; the temperature sensor, humidity sensor, differential pressure switch, pressure sensor, float switch, carbon monoxide of the building automation system sensors, carbon dioxide sensors, flow sensors, and the secondary loop feedback signals of the strong current control electric boxes of each system belong to the sensing layer and are responsible for signal collection. After the signal is collected, it is transmitted to the background through shielded twisted pair or network cable, which belongs to the transmission layer and building automation. The total monitoring platform belongs to the application layer; the ceiling-mounted ceiling speakers, wall-mounted speakers, and outdoor grass speakers of the public broadcasting system belong to the sensing layer. The transmission cables of the audio stream and the control stream constitute the transmission layer. The broadcasting workstation, the broadcasting host, the audio matrix, and the audio, the monitor, and the power amplifier together constitute the application layer; the ultrasonic detector, wireless detector, and parking guidance screen of the parking guidance system belong to the sensing layer, the twisted pair cable or network cable belongs to the transmission layer, and the parking management system server belongs to the application layer. The biggest feature of the video monitoring system is that it innovatively realizes the integration and linkage of video monitoring and conference and can manage remote equipment flexibly and effectively. The dual functions of monitoring and communication are achieved through the application of remote monitoring object recording, playback, linkage alarm, monitoring strategy formulation, emergency command, and so on. Its biggest feature is that it supports viewing video images from mobile terminals such as smart phones/tablets and supports transferring monitoring images into video conferences to realize emergency command and remote dispatching.

#### 2.1.2. Coordination Between Design and Sports Industry

The design of a folk-custom characteristic sports town must coordinate numerous intelligent building subsystems. The most important thing is to fit the theme of the town—the characteristic sports town. The slogans of some sports stars will be disseminated through intelligent media and introduced from various places. Sports categories are highly inclusive and can accept the characteristic sports industries of various places, combine local customs with local sports projects, and consider intelligent architectural design. Architectural design should achieve mutual cooperation in construction engineering and building structure. At the same time, we need to pay attention to the problem of professional cooperation in all stages of the construction project. Whether it is the feasibility study report stage, the preliminary design stage, or the construction drawing design and deepening design stage, we need to pay attention to the problem of professional cooperation at each stage of the construction project. Design works can maximize the realization of building intelligence.

#### 2.1.3. Architectural Design Should Be Consistent with Current Technology and Products

The design of intelligent buildings is inseparable from products. There are many product brands in each system, and how to choose products to realize the functions we need is also the embodiment of design art. With the continuous advancement of science and technology in our country, products in the field of intelligence have sprung up in large numbers. The variety of styles and the speed of update far leave the revision speed of the specification behind. This requires designers to go deep into the product market and understand the functions of the products on the current market. We can often see that many design drawings are technically backward, fail to keep up with the progress of product technology, and even use products that have been discontinued or eliminated on the market. Without product support, the functions of intelligent design are greatly reduced. Some designs in order to meet the needs of Party A or win the bid, regardless of what function the current product can have, exaggerated the function too much, the plan is fancy, and it is too much to say. The result is that the higher the expectation, the greater the disappointment, and the design plan cannot be implemented, and it becomes a castle in the sky. The design should not only be carried out on the basis of existing products, neither should it be advanced nor backward, but the design concept should also be moderately advanced. Human beings all have a vision for the pursuit of beautiful things. Intelligent design not only meets the existing needs but also ensures that it can meet the needs for a period of time in the future.

Intelligent media is the media that reconstructs the whole process of news information production and dissemination with artificial intelligence technology. Smart media is an ecosystem based on artificial intelligence, mobile Internet, big data, virtual reality, and other new technologies. It consists of smart media, smart media, and think tank media. The development of media convergence can be divided into three stages: all media, financial media, and intelligent media. The three stages also show different characteristics. In the all media era, media integration is a change at the physical level, while in the media integration stage, it is a chemical reaction. In the intelligent media era, it is a deep change at the genetic level.

### 2.2. Significance of Designing Folk Sports Characteristic Towns

#### 2.2.1. Promote the Economic Development of Small Towns

My country's folk culture is more produced in rural areas, and villages and towns constitute the folk culture environment. Villages in a certain area have strong similarities in terms of spatial layout and traditional customs. Such basic units can be called small towns with folk customs. However, compared to some other developed areas, the economic development of folk-custom towns lags far behind that of cities and cannot meet the needs of residents in terms of consumption or production. Therefore, the construction of sports-featured towns can well drive local economic development enables residents to better improve their lives and even get out of poverty. At the same time, they can also promote the local culture of the town. The folk-custom characteristic town has rich material and intangible cultural heritage and has a high history, The values of culture, aesthetics, society, economy, etc., spread the culture of the town to the outside world, which can further promote the cultural and economic output of the town. The planning characteristics of characteristic towns include that they can become the main body of urbanization and solve the urbanization of more people. It is more conducive to the synchronization of the four modernizations and the overall planning of urban and rural areas. It is more conducive to optimizing structure and regional balance. More conducive to ecological civilization, energy conservation, and emission reduction; Provide a characteristic life far more diverse than the city. The core competitiveness of small towns lies in the charm and vitality of characteristics.

#### 2.2.2. Intelligent Design Combined with Architectural Style

The folk sports characteristic town is based on the building integrated wiring system, and the computer network system is the core of the building's Internet of Things transmission layer architecture. This transmission layer is different from the traditional and unrelated signal transmission network. The advanced structure of the transmission layer. Once the building has this structure, it is like a highway network spread across the country. Cars at any entrance can easily reach where they want to go, because this network is shared and connected, instead of building a separate road to each place. With the building's intelligent transmission layer architecture, the addition of intelligent equipment can realize pluggable, modular, and on-demand access. For example, traditional video surveillance needs to add a monitoring probe. In addition to adding a camera, a coaxial cable must be laid to the monitoring center. It does not matter if a small-scale building is a high-rise building with dozens of floors. The amount of work required to add a probe is very large. If the building has an intelligent transport layer architecture, then this matter becomes very simple. The surveillance camera only needs to be connected to the nearest transport layer interface to easily transmit video streams, control streams, etc. to the monitoring center. The planning and design of characteristic small towns should be carried out according to the actual situation of regional development and their own core competitiveness. Agriculture, industry, and tourism are the fundamental principles. For some suburban areas close to large- and medium-sized cities, which have the conditions of convenient and fast transportation, many regional tourism elements, profound folk culture, distinctive theme characteristics, and unique landform, in the planning, design, and later construction and operation, we should vigorously combine the development of rural tourism, drive the sales of characteristic agricultural products through rural tourism and solve rural employment, provide entrepreneurial space for returning home, increase farmers' income, and build small towns with characteristics.

## 3. Research on the Design Experiment Preparation of the Folk-Custom Characteristic Town

### 3.1. Experimental Method

The main methods used in this paper are the total variation method of the unary function and the sum of squares of variation. The unary function total variation method is a relatively simple measurement method. It has been implemented in many practical applications, and the measurement principle is as follows.

1. Unary function total variation method

The total variation of a function *f*(*x*) in a certain interval [*a*, *b*] is the sum of the variation range of the function value, and *D* represents the total variation; then, there is

(1) $$\begin{array}{c} D=\overset{n-1}{\underset{i=1}{\sum }}abs\left(f\left(x_{i+1}\right)-f\left(x_{i}\right)\right). \end{array}$$

Among them, *a* = *X*1 < *X*2 < *X*3 < ⋯<*Xn* = *b* is a division of the interval [*a*, *b*], and the length of the subintervals [*Xi*, *Xi* + 1] all tend to zero.

(2) Sum of squares of variance

For the convenience of formula derivation, the sum of squares of variation can be used. In this article, the sum of squares of variance of a function *f*(*x*) in a certain interval [*a*, *b*] is represented by D2, and it is specified:

(2) $$\begin{array}{c} D^{2}=\overset{n=1}{\underset{i=1}{\sum }}\left(f\left(x_{i+1}\right)-f\left(x_{i}\right)\right). \end{array}$$

Variance is a measure of the degree of dispersion when probability theory and statistical variance measure random variables or a group of data. In probability theory, variance is used to measure the deviation between random variables and their mathematical expectations (i.e., mean). Variance in statistics (sample variance) is the average of the square value of the difference between each sample value and the average of all sample values. In many practical problems, it is of great significance to study the variance, that is, the degree of deviation. Variance is a measure of the difference between the source data and the expected value.

### 3.2. Experimental Data Collection

This paper establishes a mathematical model based on the Internet of Things technology and uses a questionnaire survey method to collect the willingness of 324 volunteers, analyze the collected data, and obtain the corresponding survey results through analysis and comparison, and analyze the objective function and calculate the optimal configuration that meets the requirements. The classification of questionnaire survey method is divided into self-administered questionnaire survey and substitute questionnaire survey according to the different respondents. The self-administered questionnaire survey can be divided into newspaper questionnaire survey, postal questionnaire survey, and delivery questionnaire survey according to different ways of questionnaire transmission. The surrogate questionnaire can be divided into interview questionnaire and telephone questionnaire according to the different ways of talking with the respondents.

## 4. Research on the Experimental Preparation of the Folk-Custom Characteristic Sports Town

### 4.1. Analysis of Sports Preference

This article conducts a statistical analysis of the collected data through interviews with 200 volunteers. This data collection is collected from different groups of people. There is no preference and can greatly avoid the influence of external factors.

It can be seen from Table 1 and Figure 1 that people who like ball games account for the largest proportion, with 156 people accounting for 48.15%. This shows that about half of the people like ball games, which proves that ball games should be used in folk sports towns. Sports are the main body, and other sports are supplemented. At the same time, in order to reflect compatibility, other types of sports should also be included, but they should not have a large proportion, or it will be counterproductive. Track and field sports are ranked second. There are 73 people accounting for 22.53. There are more people in China who like to run to keep fit. Running is also suitable for men, women, old and young, and people of all ages, which deserves attention.

### 4.2. Comparative Analysis of Ball Game Preferences

In order to verify people's preference for balls in ball games, we conducted statistics again among the 156 investigators who chose ball games to collect and analyze data on several traditional ball games to analyze the most popular balls.

As shown in Figure 2, the most popular ball sports are basketball and football. This may be because they are also the most recognized and popular ball sports in the world. At the same time, there are some internationally famous NBA stars and World Cup football stars. The influence of athletes cannot be ignored. The industrial influence brought by these stars is huge, and they are greatly satisfied with people's spiritual pursuits. Therefore, this also inspired this research. In China, attention should be paid to the development of the two most popular ball games, basketball and football. 96 of 156 people chose basketball and football, accounting for more than 60%. Therefore, strengthening the construction of football and basketball ball games is very meaningful.

### 4.3. Analysis of Support Rate of Folk Sports Towns

In order to understand the surveyors' folklore sports towns, a total of 324 surveyors were statistically analyzed for their support rate. The surveyors can choose four options, “very support,” “comparative support,” “general support,” and “not support,” and use this to analyze the public's views on sports towns.

As shown in Table 2 and Figure 3, only 48 of the 324 people expressed disapproval, accounting for 14.81%. This shows that most people hold a supportive attitude, indicating that sports culture still occupies a relatively important position in people's hearts. Some people's emphasis on the development of sports is of great significance to the development of sports culture in our country. More than one-third of 123 people expressed their supportive attitude, indicating that the folk-custom sports town has great prospects for development. The main contents of folk sports are as follows: national traditional sports with a long traditional history, national color, and strong folk culture; sports inherited by ethnic minorities; in different historical periods, folk sports activities are widely spread among the people through national exchanges, digestion, and absorption.

### 4.4. Analysis of the Degree of Understanding of Intelligent Building Theory

The application of smart buildings in our country has not been popularized in various regions, so people have more or less knowledge of the concept of smart buildings. Therefore, it is necessary to conduct questionnaire surveys to understand their understanding of smart buildings.

As shown in Figure 4, 48.15% of the respondents indicated that they did not know much about smart buildings, indicating that the concept of smart buildings is less popular in people's lives, and people still know very little. The construction is very meaningful. Among the investigators who fully understand the theory of intelligent buildings, only 15 people and about 4.63 people said that they have complete understanding. The construction of intelligent building towns can greatly spread the concept of intelligent buildings and make people's lives more interesting. Intelligent development.

## 5. Conclusions

This article uses intelligent building technology to analyze the folk-custom characteristic sports town, introduces the intelligent design viewpoints and design significance of the folk-custom sports characteristic town, and collects and analyzes the survey data of 324 investigators, including the preferences of various sports items. Analyze and further analyze the most popular ball games. At the same time, compare the previous proportions of different ball games. It is concluded that the ball sports are the most popular and have broad prospects, combined with intelligent architectural design, to integrate modern smart home smart technology and connect them in series through the Internet of Things technology. Since the Internet of Things has many advantages and easy operation, the country puts the development of the Internet of Things first. In addition to certain improvements in information transmission, the Internet of Things has a lot of room for realizing the intelligentization of folk-custom towns. In terms of power transmission, consumption, and power management, it has changed the passive form of the past. The one-way transmission is a two-way transmission, which greatly improves the efficiency of power transmission, and at the same time, the management of power will become more convenient. Nowadays, in the development concept of the folk-custom characteristic sports town, the Internet of Things is introduced into the intelligent construction to realize the intelligent development of the town.

## Figures and Tables

**Figure 1:** Sports preference analysis.

**Figure 2:** Comparative analysis of ball game preferences.

**Figure 3:** Analysis of support rate of folk-custom sports towns.

**Figure 4:** Analysis of the degree of understanding of intelligent building theory.

**Table 1:** Sports preference analysis.

Sports items	Number of people	Percentage (%)
Ball	156	48.15
Track and field	73	22.53
Diving	25	7.71
Weightlifting	46	14.20
High jump	24	7.41

**Table 2:** Analysis of support rate of folk-custom sports towns.

Support rate situation	Number of people	Percentage (%)
Very supportive	123	37.96
More support	85	26.24
General support	68	20.99
Not support	48	14.81

## Data Availability

The data underlying the results presented in the study are available within the manuscript.
